This article has been retracted.

# Using Decision Tree Classification and AdaBoost Classification to Build the Abnormal Data Monitoring System of Financial Accounting in Colleges and Universities

**DOI:** 10.1155/2022/1467195

**Published:** 2022-09-16

**Authors:** Yan Jiang

**Affiliations:** Shandong Sport University, Jinan, China

## Abstract

In order to better solve the problems of low efficiency, large consumption of human resources, and relatively low degree of intelligence in the abnormal data monitoring system of financial accounting in colleges and universities under the background of current accounting computerization, this article takes data mining and neural network algorithm as the technical basis to build the abnormal data monitoring system of financial accounting in colleges and universities. This article uses data mining algorithm and neural network analysis technology to process the original accounting information of colleges and universities, effectively eliminate invalid data, retain valuable data, and improve the detection efficiency of abnormal accounting data. The system test results show that the accuracy of identifying 50 abnormal situations in the original accounting data of colleges and universities is more than 90% by using data mining and neural network model.

## 1. Introduction

Accounting computerization is becoming more and more popular in the financial accounting application of enterprises in our country. Accounting computerization gradually replaced the original financial accounting software. With the help of computer network technology and information processing technology, the efficiency of financial accounting information processing can be further improved, as shown in Figure 1 [1]. But with the development of accounting computerization, the enterprise accounting process also began to expose some problems. For example, the original data processing ability is relatively poor, and the identification of abnormal data is relatively difficult. After all, traditional accounting computerization still requires manual input of financial data information into the system and then use simple logic and manual audit to judge whether there is abnormal data. This workflow is less efficient, and data processing accuracy is lower. Therefore, based on a comprehensive review of the shortcomings of traditional accounting algorithms, this study uses data mining and neural network algorithm to build a more scientific and efficient accounting abnormal data monitoring system and verifies the feasibility of the algorithm model through system testing [2].

## 2. Literature Review

The current research focuses on qualitative and quantitative analysis methods. Some scholars believe that quantitative analysis should be adopted for early warning of financial risks of enterprises. Through the construction of data model, the standard of risk degree is determined, and the purpose of early warning is finally achieved [3]. Some scholars take the model as the breakthrough point, propose how to establish the enterprise financial early warning system, and design the process and content of the system; its purpose is to reduce the damage caused by financial risks to enterprises [4]. When monitoring problems, managers can take decisive action against the relevant data and quickly find countermeasures to curb the occurrence of financial crisis. Chen et al. [5] established financial risk early warning mechanism by establishing unitary discrimination model and multivariate discrimination model. The study of internal control of enterprises will be introduced into the analysis of financial early warning, and the strength of working capital management of the company will be increased so as to gradually reduce the cost of enterprise financial risk and finally realize the purpose of early warning and effective management of enterprise financial risk [5]. Li et al. [6] introduced the relevant theoretical knowledge points of internal control in detail and then introduced the risk early warning system in detail. The financial indicators of enterprises are determined from three aspects, and a linear financial risk warning model is finally constructed according to the critical value of financial indicators [6]. Zhan et al. [7] proposed various main financial risk evaluation methods and models, namely, univariate decision model, multiple linear evaluation model, and comprehensive scoring method. According to the analysis of the characteristics of these three methods, the multiple linear evaluation model is obtained, namely model [7]. The model can objectively and accurately judge the financial risks of enterprises and put forward solutions according to the shortcomings of the model itself. Yin et al. [8] studied the financial risks of enterprises by taking cash flow index as the early-warning variable of financial risks and built a model on this basis. The expected cash flow and risk cash flow are used as independent variables to construct a binary early warning model. Finally, enterprises and nonenterprises are selected as empirical samples [8]. According to the research results, the model can better reflect the cash flow of the enterprise, and the early warning model can play a role in the early warning of enterprise finance. Gong et al. [9] believe that it is not accurate to analyze the financial statements of enterprises by a single quantitative method in the current financial early warning system. Because the situation of different enterprises is more complex, the use of a single quantitative analysis cannot fully reflect the existence of enterprise financial risk. Only by combining quantitative and qualitative analysis can an enterprise's financial crisis situation be more accurately reflected [9]. Jalal and Ali [10] considered that a single quantitative analysis was not consistent with the situation of the enterprise and might even have a contradictory effect. They emphasized that qualitative analysis plays a pivotal role in the early warning of corporate financial risks, especially the important role of cash flow indicators [10]. It is proposed that the analysis of financial crisis warning should combine qualitative analysis with quantitative analysis.

## 3. Data Mining Algorithm Based on Deep Neural Network

### 3.1. Decision Tree Classification Algorithm

The key issue in distribution is how to develop good training models. The logging algorithm is less complex and has more isolation. At the heart of the woodworking algorithm is the reduction of uncertainty after partitioning [11]. The specific steps are as follows: divide the data gain of the sample set *S* (*S*, *A*) by the property a and subtract the entropy of the sample set S from the entropy of the sample set.

(1) $$\begin{array}{c} Gain\left(S,A\right)=Entropy\left(S\right)-{Entropy}_{A}\left(S\right). \end{array}$$

If *A* is a discrete value with a difference of *K*, then *A* divides *S* into a subset of *K*. {*S*_1_, *S*_2_, *S*_*k*_} according to the *k* values, and the entropy value of data set *S*is divided by using *A* as follows:

(2) $$\begin{array}{c} {Entropy}_{A}\left(S\right)=\overset{k}{\underset{i=1}{\sum }}\frac{\left|S_{i}\right|}{\left|s\right|}Entropy{\left(S\right)}_{i}\text{.} \end{array}$$

If *A* is a continuous value, then in ascending order of the value of *A*, the midpoint of each pair of adjacent values is regarded as the possible splitting point, and each possible splitting point is calculated as follows:

(3) $$\begin{array}{c} {Entropy}_{A}\left(S\right)=\frac{\left|S_{L}\right|}{\left|s\right|}Entropy\left(S_{L}\right)+\frac{\left|S_{R}\right|}{\left|s\right|}Entropy\left(S_{R}\right)\text{.} \end{array}$$

Then, the information gain rate is

(4) $$\begin{array}{c} GainRatio\left(S,A\right)=\frac{Gain\left(S,A\right)}{SplitInformation\left(S,A\right)}\text{.} \end{array}$$

The split information is

(5) $$\begin{array}{c} SplitInformation\left(S,A\right)=\overset{k}{\underset{i=1}{\sum }}\frac{\left|S_{i}\right|}{\left|S\right|}\log_{2}\frac{\left|S_{i}\right|}{\left|S\right|}\text{,} \end{array}$$

where *S*_1_ ~ *S*_*k*_ stands for dividing attribute *A* into*k* different subsets and |*S*| is the size of sample set [12]. For all nonleaf nodes, the misclassification rate after pruning is counted. Its estimation usually refers to the upper limit of the confidence interval. For the immediate confidence threshold *ɑ* (generally 0.25 by default), the number of errors follows the binomial distribution:

(6) $$\begin{array}{c} \mathrm{Pr}\;\left(\frac{\left|f-q\right|}{\sqrt{q\left(1-q\right)/N}}\geq U_{1-\alpha }\right)=\alpha \text{.} \end{array}$$

*N* is the total number of samples, *E* is the number of incorrect classifications in the sample *N*, then *f* = *E*/*Nf* is the observed error rate, and *q* is the actual error rate. Use the following formula (7) to make the standard deviation of confidence ɑ:

(7) $$\begin{array}{c} z=1-U_{1-\alpha }. \end{array}$$

Then, the confidence upper limit of *q* can be calculated, and the node error rate *e* can be estimated by this upper limit:

(8) $$\begin{array}{c} e=\frac{f+\left(z^{2}/2N\right)+z\sqrt{\left(f/N\right)-\left(f^{2}/N\right)+\left(z^{2}/4N\right)}}{1+\left(z^{2}/N\right)}\text{.} \end{array}$$

Therefore, pruning can be determined by the size of *e* before and after pruning [13].

### 3.2. AdaBoost Classification Algorithm

Boosting, as AdaBoost, is the most typical algorithm of Boosting family, and Boosting, as a meta-algorithm framework, can basically be combined with all data mining algorithms to improve classification accuracy with good results [14]. The core process of ensemble learning AdaBoost.*m*1 algorithm suitable for multiclassification is given as follows:

Input: Sample set:

(9) $$\begin{array}{c} S=\left\{\left(x_{1},y_{1}\right),\left(x_{m},y_{m}\right)\right\},y_{i}\in Y=\left\{1,2,k\right\}\text{.} \end{array}$$

In the above formula, *m* is the number of samples, *k* is the number of decision categories, the number of iterations *T*, and the data set S is used as input. For each sample (*x*_*i*_, *y*_*i*_) ∈ *S*, the initial weight distribution is as follows:

(10) $$\begin{array}{c} D_{1}\left(x_{i},y_{i}\right)=\frac{1}{m}\text{.} \end{array}$$

(1) Start *T* cycle iterations:
  (11) $$\begin{array}{c} fort=1,2,T\text{.} \end{array}$$
(2) Under the current distribution *D*_*t*_, the classification rules of round *t* are constructed by using the weak classifier (decision tree classification algorithm in this article) as follows:
  (12) $$\begin{array}{c} h_{t}:X⟶Y\text{.} \end{array}$$
(3) Calculate the misclassification rate of weak classifier *h*_*t*_ as follows:
  (13) $$\begin{array}{c} \varepsilon_{t}=\overset{m}{\underset{i=1}{\sum }}D\left(x_{i},y_{i}\right)\left[h_{t}\left(x_{i}\right)\neq y_{i}\right]\text{,} \end{array}$$
*D*(*x*_*i*_, *y*_*i*_)is the weight of the sample in the *i*th cycle.
(4) Calculate the classification weight of weak classifier in round T as follows:
  (14) $$\begin{array}{c} \beta_{t}=\frac{\varepsilon_{t}}{\left(1-\varepsilon_{t}\right)}\text{.} \end{array}$$
(5) Update the weight vector of the sample as follows:
  (15) $$\begin{array}{c} D_{t+1}\left(i\right)=\frac{D_{t}\left(i\right)\beta_{t}^{1-\left[h_{t}\left(x_{i}\right)\neq y_{i}\right]}}{Z_{t}}\text{.} \end{array}$$
(6) After *T* times of cyclic iteration, a strong classifier combination is formed as follows:
  (16) $$\begin{array}{c} H\left(x\right)=arg\max_{y\in Y}\left(\overset{T}{\underset{i=1}{\sum }}\log\frac{1}{\beta_{t}}\left[h_{t}\left(x\right)=y\right]\right)\text{.} \end{array}$$

Among them, if the expression in is true, it is 1; otherwise, it is 0.

Therefore, the abnormal traffic classification detection problem in this chapter can be described as follows: let *R*={*R*_1_, *R*_2_, *R*_*m*_} represent the traffic set of *m* consecutive unit statistical Windows, *R*_*i*_={*S*_1_, *S*_2_, *S*_*n*_} represent the traffic set of the *i*th unit statistical window, and*S*_1_ to *S*_*n*_ represent the *n*-dimensional traffic characteristics in the unit statistical window. Let *T*={*T*_1_, *T*_2_, *T*_*m*_} represent the network traffic detection results in *m* unit statistical windows. The core idea of abnormal traffic classification detection is to obtain the mapping of traffic sets in each unit statistical window to network status results. *F* : *R*⟶*T*, *F*(*R*_*i*_)=*T*_*k*_ indicates that the detection result of the *i*th unit statistical window is normal or abnormal, where *i*=1*n*, *k*=1*m*. In this article, AdaBoost algorithm is used to further improve the performance of the decision tree and construct a strong classifier model to find the mapping *F* [15].

## 4. Design and Implementation of Abnormal Accounting Information Detection System Based on Data Mining

### 4.1. System Framework

The general structure of the system is shown in Figure 2. As shown in the figure, the system is divided into four stages: product analysis stage, data processing stage, standardization processing stage, result and early warning stage [16]. The purpose of interpretation is always financial. This line will guide the data in the financial process which always follow the data, make the data write channel, and carefully monitor it. Then comes the data processing part, which uses data mining technology to process the obtained original data. The purpose of data preprocessing is to make the data easier to process by data mining models. Data quality can have a significant impact on data mining models. It can be argued that data and features already set an upper limit on the knowledge that can be acquired and that data mining models only approximate the upper limit. Various preprocessing techniques have been invented to make the data meet the input requirements of the model, improve the relevance of the prediction target, and make the optimization step of the model easier. It is basically divided into three modules: data collection, data preprocessing, and data encoding [17]. The initial data preprocessing module includes removing special equipment, assembling relevant equipment, completing incomplete results, and data samples so as to convert old data into usable data. The old data can be converted to useable data [18]. The data encoding module is usually responsible for encoding the sample data so that all the data can be accessed directly from the intelligent algorithm that forms the basis of the intelligent identification section. Next is part of the analysis process. Once completed, financial data will be used to train intelligent strategies. The last section is the results and report section, which uses a plan to analyze financial information, draw up erroneous data, report, and provide financial advice to the financial statements, so it creates a closed loop [19].

### 4.2. Data Acquisition and Data Processing

The system is divided into two parts: data collection and data processing. The special procedures required to perform in this system are as follows[20].

#### 4.2.1. The Realization of Data Acquisition

The information required by the system is usually of three types: information such as name, gender, age, position, hours of service, position, job, average monthly income, and other information. This information can be obtained directly from the human resources department and financial institutions through the company's internal network. The second category includes rewards and incentives, including seasonal bonuses, final year bonuses, all types of bonuses, grants, and other information. Such information can be obtained directly from the departmental records because the department usually provides the information as a function. The third category includes payment information for travel business, which usually includes location, time, type, delivery time, and various invoices and fees. This information is usually provided by individuals and verified by office administrators [21]. As network technology has evolved, the collection of this information has become more effective.

#### 4.2.2. The Realization of Data Processing

Data processing can be divided into two parts: preprocessing and coding. The following two sections describe the use of these two sections.

First: the realization of data preprocessing.

The basic data preprocessing process is shown in Figure 3.

Figure 3 shows the issues that need to be addressed in advance of the data and solutions. The following procedure is shown as an example in Python.

*(1) Unique Attribute Processing*. The special refers to features that can identify a particular feature, such as name and function number but do not affect the identification of unusual data and can be removed immediately. The instructions removed from Python are as follows: data.drop (‘feature_name', axis = 1)

Or

data.drop (‘feature_name', axis = 0)

Use this command to delete all file rows or columns from the Feature_name property. Axis = 1 means minus 1 line, and axis = 0 means minus 1 line.

*(2) Processing of Missing Data*. Missing value processing steps are as follows: (1) find the missing value position and (2) filling of missing values [22]. The Pandas library is used to search for the lost value of a given feature. It is used to search for the lost value of a given feature.

position = pandas.isnull (feature_name);

This function returns the default value of the missing value in the Feature_name property that can be used to make the missing value.

*(3) Merge Related Attributes*. For the data of a specific function, you can combine the relevant data into one data and use data processing to delete the other data. Reduce the size of the calculation to achieve the goal of data aggregation [23].

For Python, the process is as follows: data [“feature_name1”]

 = data [“feature 1”] + data [“feature2”]

data.drop (‘feature2', axis = 1)

The first sentence of the program adds two lines of data items, feature 1 and feature 2, and the second sentence acts as a removable after merging item. For example, years of service, years of entry, and related information may come together. During this time, preprocessing of old data is accomplished in order to turn old data into nonuseable and only useable data.

Second: the realization of data coding.

File encoding is the process of converting specialized data from easily understood data into easy-to-machine-readable data. Based on data encoding, it can be divided into nonencoding files and further processing files. The special operating procedures are as follows.

*(1) For Discrete Data*. One or more character separations can be grouped into classes within a single product, and each class can be separated using the One_Hot encoding process. In Python, you can easily use the panda science library.

*(2) For Continuous Data*. To make it easier to understand the extension data, the extension data can first be sorted into sections and then access the extension using the One_Hot format. In Python, you can compile extended files using custom functions. The custom operation call format is as follows: data.apply (function, axis = 1)

As an example of the dichotomous method, the method of continuous data separation was introduced.

  def function (DataFrame):
  feature = data [“feature_name”]
  if pandas.isnull (feature):
  return “error”
  elif feature < Threshold:
  return “class1”
  else:
  return “class2”

The above operations continuously separate the Feature_name Feature file from the Specific_name by default. Data can be encoded using discrete encoding.

#### 4.2.3. Implementation of Identification Process and Output

The definition of external data can be understood as data sharing, for example, all data can be divided into natural and non-natural data, local data, unreliable data, and abnormal data. The basic distribution process is as follows: Support Vector Machine (SVM) is used to develop procedures for estimating and distributing e-commerce microblogging gossip and ordering quantity. SVM method is used to measure and distribute network risks, personal credit, and daily state stress, and SVM method is used to distribute state signals and detect errors [24]. Currently, the SVM algorithm has been widely used for application distribution, but it is still difficult to implement large instruction models. The classical support vector machine algorithm only provides two-class classification algorithms, but in the practical application of data mining, it is generally necessary to solve multiclass classification problems. It can be solved by a combination of multiple second-class support vector machines. There are mainly one-to-many combination mode, one-to-one combination mode, and SVM decision tree; then, it is solved by constructing a combination of multiple classifiers. The main principle is to overcome the inherent shortcomings of SVM and combine the advantages of other algorithms to solve the classification accuracy of multiclass problems. For example, combined with rough set theory, a combined classifier for multiclass problems with complementary advantages is formed. Providing an environmentally friendly application for monitoring financial variables, the system uses BP neural network as a technology, with the most flexible and scalable process. The procedure for doing this is as follows.

1. The number of input functions and the encoding bits for each feature can determine the number of neurons in the input layer of the neural network.
2. Determination of the middle layer.
3. Output layer design.

Currently, neural networks have been established and data completion is used to train neural networks. The training is shown in Figure 4.

Finally, the prepared neural network is used to monitor and analyze abnormal financial data, identify normal and abnormal financial data, and supply abnormal financial data to the financial system.

### 4.3. Abnormal Data Detection System Architecture

The whole system consists of four modules: traffic acquisition and analysis, data preprocessing (feature extraction engine, dimension reduction algorithm), data storage, and abnormal traffic classification and detection. The overall design architecture of the system is shown in Figure 5.

Software must be mature and modular. Maturity is the use of accepted technology to ensure system performance and viability; software modularization refers to software that is reasonably divided into relatively independent modules, which is conducive to software system maintenance and upgrade. The traffic anomaly detection system in this article uses MVC-based multilayer software design pattern. In this design mode, the business logic, data model, and interface display are separated effectively so that the parallel operation and computing ability of the system are improved, and the overall performance of the system is optimized. It is mainly divided into performance layer, business layer, and data layer. The specific technical architecture of the system in this article is shown in Figure 6.

Abnormal data monitoring requires scientific detection of abnormal network flow of the computer financial accounting system. The development environment of each module of the flow anomaly detection system is MyEclipse 10, using Java, MySql 5.5 as database, and Windows7 as operating system. In order to simplify the development, related JAR packages in Weka are introduced to support the abnormal traffic classification module, and secondary development is carried out on this basis. This section will describe the realization idea of each module and the core data structure in detail. Jpcap does not complete the control of the data link layer in the real sense in Java. Jpcap ultimately calls winpcap at the bottom layer so as to provide Java with an interface to access the resources at the bottom of the network, thus having the advantage of platform independence [25]. Winpcap is an excellent network data acquisition and network research framework, including filter, packet.dll, and wpcap.dll. The main function of winpcap is to send and receive raw data packets independently of host protocols such as TCP-IP. That is to say, winpcap cannot block, filter, or control the sending and receiving of packets from other applications, it just listens for packets transmitted on the shared network. The specific process of capturing network packets is shown in Figure 7:

In this article, only the stream records that have not been terminated in the history window are maintained in the current window rather than all previous stream records. If a stream has not been terminated for more than 30 seconds, it is forcibly terminated. The purpose of this is on the one hand to reduce resource consumption and release memory in time. On the other hand, the previous statistical window may contain the flow record information in the next statistical window. According to the required statistics, add counters in corresponding state nodes to count the number of packets in different states. The core ideological process of feature extraction in this article is shown in Figure 8:

Abnormal traffic classification module is the core module of the whole system. The feature samples extracted by the feature extraction engine module in the statistical window will pass through the traffic classification module to give classification results. In P2P traffic identification module, a decision tree classifier is constructed, and in abnormal traffic classification module, AdaBoost algorithm is used to further improve it into a strong classifier. The main reason is that the identification accuracy of P2P traffic identification module is relatively high, and there is no need to further improve it into a strong classifier.  Figure 9 shows the processing flow of abnormal traffic classification module in this article:

The whole abnormal traffic classification consists of two processes, offline training and online classification. Since it is necessary to do secondary development on the basis of relevant JAR packages in Weka, it is necessary to understand its underlying encapsulation of relevant algorithms. The construction of weak classifier is the core process in P2P traffic identification and abnormal traffic classification. In the offline training stage, parameter setting and model construction are usually completed. In the offline training phase, parameter setting and model building are usually completed. The server sets a sufficient number of reference points in the area of interest, and the mobile device measures its Wi-Fi fingerprint at each reference point, that is, the received signal strength value of the surrounding Wi-Fi APs, and then, the server collects the fingerprint information of each reference point, stores it in the fingerprint database, and builds fingerprint map. The decision tree algorithm is separately encapsulated as the class J48. First, the object needs to be instantiated, and then, the core parameters of the algorithm are set by the setOptions () function, and the classification model is established by the buildClassifier () function. Relevant parameters of decision tree training model are stored in String array [26]. The core parameters are as follows: −*c* represents the confidence threshold of pruning, −*u* decision tree does not pruning, −*m* represents at least the number of instances on the leaf node, and −*r* represents the pessimistic error pruning method (REP) as the pruning algorithm. The decision tree in this article will be pruned using REP. The level of confidence in the pruning is 0.25, and the number of cases on the leaf nodes is not less than 2.

## 5. System Experiment Verification

### 5.1. The Experiment A

In this article, a strong classifier model based on AdaBoost and decision tree data mining algorithm is constructed to classify abnormal traffic [27–35]. Through the analysis of feature selection algorithm in this article, some redundant features and features that do not have the ability to distinguish abnormal traffic are removed [36]. According to every 1000 TCP packets as a unit statistical window, the following six attributes are selected to construct abnormal traffic classification detection model. The specific meanings are also analyzed in depth in this chapter. The names and descriptions of characteristic attributes are shown in Table 1.

Valuable field information of network data packets in Pcap file was extracted through the program and stored in the database. A total of 26,236 valid sample data required for the modeling experiment were generated using traffic organization and logical calculations as shown in Table 2.

In the simulation analysis under Weka, the performance of the model is evaluated by cross-validation of ten folds. In this article, traffic is classified into three categories: Normality, DDoS, and Scan. Classification accuracy and false positives are mainly used to measure the performance of classification models. In addition, performance comparisons are made with Naive Bayes (NB), SVM, and C4.5 models of the decision tree. The details of the three types of classifications are shown in Figure 10.

 The detailed performance pairs of each algorithm are shown in Table 3. The AdaBoost algorithm used in this article has a significant effect on improving the weak classifier C4.5, which can only be seen to be better than the C4.5 algorithm. Compared to the three comparative algorithms, it has advantages in terms of classification accuracy and overall classification accuracy. This can to some extent effectively address the current situation where the detection rate of the current abnormal flow detection system is low and the false-positive level is high. NB classification model is established on the basis of the independence of each attribute feature and follows the Gaussian distribution, so it is difficult to meet, so the recognition effect is not ideal, and the recognition rate is lower than C4.5 and SVM. SVM modeling time is too long, which is not conducive to real time. C4.5 does not depend on the prior probability of the training data, which can avoid the disadvantage caused by the imbalanced data distribution. It is simple, efficient, and has significant advantages in analyzing and processing large-scale data. Since the AdaBoost algorithm is used to improve the performance of the weak classifier, this paper verifies through the simulation of the sample, when the number of iterations is 8, the classification effect is the best. As shown in Figure 11, the values for the performance evaluation of weak classifiers (incorrect classification level and weight) vary depending on the number of iterations. At each iteration, the sample weight distribution is continuously adjusted by the percentage of incorrect classification, and it can be seen that the percentage of incorrect classification of the classifier is continuously decreasing. The higher his weight, the more important it is to make the final decision.

Aiming at the existing network data, the influence of packet number in unit statistical window on classification accuracy is also studied. Finding the optimal size of unit statistical window is of great significance to abnormal traffic detection system. Too large statistical window is not good for real-time performance, and too small statistical window has great error for accurately describing abnormal traffic characteristics. When the number of packets in the unit statistical window increases from 500 to 1200 with an increasing gradient of 100, the overall classification accuracy of the classifier changes as shown in Figure 12:

It can be seen from Figure 12 that, within a certain range, classification accuracy increases with the increase of the number of packets in the statistical window. When the number of packets in the unit statistical window is between 900 and 1000, the classification accuracy reaches the maximum value and then reaches a relatively stable state.

### 5.2. The Experiment B

To test the effectiveness of the system, select 500 types of business travel invoice compensation records for a particular enterprise, including 50 abnormal data as initial data. The selected system properties are as follows: the city of business trip is divided into 3 categories, the duration of business trip is divided into 3 categories, the difference of arrival and departure time of adjacent vehicles is divided into 2 categories, and the average daily reimbursement amount is divided into 3 categories. The output is of two types: abnormal 0 and normal 1. Because there is a small amount of abnormal data in the system, 400 abnormal data are generated in the data set according to the exception rule and then added to the data set. Relevant parameters of neural network design are shown in Table 4.

900 data were randomly divided into two groups: 800 training sets and 100 neural network training test sets. The final test results show that 51 of 54 normal data and 45 of 46 abnormal data are correctly identified in the test set, and the comprehensive recognition success rate is 96%. The neural network model is used to identify 50 abnormal data in the original data, 45 of which are correctly identified, and the accuracy rate is 90%.

## 6. Conclusion

With the development of artificial intelligence technology, the integration of artificial intelligence technology and accounting theory to improve the accuracy and efficiency of asset management has become a hotspot of research. Some studies have highlighted the need for a combination of artificial intelligence for the future development of the accounting industry and suggested the use of artificial intelligence, accounting theory, and the practice of integrating smart accounting schemes. It also proposes to do more research on accurate monitoring and forecasting of stock market wealth and to create a dynamic system of early financial warning based on artificial intelligence technology. Some scholars have used in-depth learning and networking to create internal intelligent audit systems based on financial sharing models. Many of these studies focus on financial theory analysis, which only identifies financial models, but have no clear understanding and are therefore ineffective. To address this issue, this paper focuses on the analysis of data and the use of algorithms for tracking and analyzing various financial information in the neural network. There are certain standards and ways in which financial information imbalances can be addressed. This document provides a new system for monitoring and analyzing financial variables based on data mining and neural networks and provides detailed models for addressing data underutilization, integrates accounting and knowledge, recognizes variable-based business travel business fees, analyzes data, explains early warnings, and identifies 50 differences in initial data from colleges and universities using data mining and psychology. It is a network model with more than 90% accuracy. System performance is guaranteed. At the same time, the system still has some defects, and often the training time of the neural network is long, and the initial value of the neural network is not able to provide guidance. Optimizing the initial cost of the network and eliminating network inconsistencies will be the focus of further research.

## Figures and Tables

**Figure 1:** Accounting anomaly data monitoring.

**Figure 2:** Overall framework of the system.

**Figure 3:** Data pretreatment.

**Figure 4:** BP neural network training process.

**Figure 5:** Overall design architecture of the system.

**Figure 6:** Software technical architecture.

**Figure 7:** Jpcap capture packet flow chart.

**Figure 8:** Core thought flow diagram of feature extraction engine.

**Figure 9:** Abnormal traffic classification module.

**Figure 10:** Comparison of classification accuracy of various algorithms.

**Figure 11:** Schematic diagram of AdaBoost algorithm performance improvement.

**Figure 12:** Influence of number of packets in unit statistical window on classification accuracy.

**Table 1:** Characteristic attributes and description.

Attribute name	Character description
Single_Flow_Rate	Percentage of single packet flow in unit statistics window
Proteco_lSymmetry	Ratio of THREE-way handshake SYN packets to ACK packets in the unit statistics window
Rst_Packet_Num	Unit number of abnormal RST packets in the statistics window
TTL_Anomaly_Value	Unit number of network flows containing the right abnormal TTL value in the statistics window
Service_Rate	Service rate in unit statistics window
Dest_IP_Entropy	Entropy of the target IP address in the unit statistics window

**Table 2:** Description of training samples.

Flow type	Sample size (item)
Normal flow	14880
DDoS attack abnormal traffic	7725
Scanning abnormal traffic	3631

**Table 3:** Performance analysis of each algorithm.

Algorithm name	Modeling time (s)	The rate of false positives (%)	Overall classification accuracy (%)
NB	0.06	1.9	93.72
SVM	5.69	1.39	94.63
C4.5	0.26	1.2	95.76
AdaBoost + C4.5	1.39	0.86	98.60

**Table 4:** Parameter Settings of neural network.

Parameter	Values
Number of neurons in the input layer	11
Number of neurons in output layer	2
Number of hidden layer neurons	25
Training goal	0.01
Learning rate	0.1
Output neuron function	Logsig

## Data Availability

The data set can be obtained from the author upon request.
